# The impact of financial contagion on real economy-An empirical research based on combination of complex network technology and spatial econometrics model

**DOI:** 10.1371/journal.pone.0229913

**Published:** 2020-03-06

**Authors:** Xiurong Chen, Aimin Hao, Yali Li

**Affiliations:** School of Economics, Zhengzhou University of Aeronautics, Zhengzhou, China; Shandong University of Science and Technology, CHINA

## Abstract

This study presents financial network indicators that can be applied to inspect the financial contagion on real economy, as well as the spatial spillover and industry aggregation effects. We propose to design both a directed and undirected networks of financial sectors of top 20 countries in GDP based on symbolized transfer entropy and Pearson correlation coefficients. We examine the effect and usefulness of the network indicators by newly using them instead of the original Dow Jones financial sector as explanatory variables to construct the higher-order information spatial econometric models. The results demonstrate that the estimated accuracies obtained from both the two networks are improved significantly compared with the spatial econometric model using the original data. It indicates that the network indictors are more effective to capture the dynamic information of financial systems. And meanwhile, the accuracy based on the directed network is a little higher than the undirected network, which indicates the symbolized transfer entropy, i.e. the directed and weighted network, is more suitable and effective to reflect relationships in the financial field. In addition, the results also show that under the global financial crisis, the co-movement between financial sectors of a country/region and the global financial sector as well as between financial sectors and real economy sectors is increased. However, some sectors in particular Utilities and Healthcare are impacted slightly. This study tries to use the financial network indicators in modeling to study contagion channels on the real economy and the industry aggregation effects and suggest how network indicators can be practically used in financial fields.

## 1. Introduction

The complex network theory has been rapidly applied to various fields such as biology, physics, medicine and especially finance since it greatly promotes the development of economic physics, provides people with deeper understanding on complex financial system[1]. As we know, with the continuous development of the modern financial industry, the increasing participants in the financial market has gradually evolved into a complex system formed by the participation of multiple entities such as governments, financial institutions, corporate organizations, and individuals, with infinitely extended connections in time and structure. Faced with such a complicated financial system, it has become extremely difficult to analyze the contagion between financial markets and real economy. While the traditional financial theory based on the hypothesis of idealization, formalism, and linear singularity, is inconsistent with the complexity of the actual financial system, i.e. this complexity has caused traditional financial theory to encounter insurmountable obstacles. However, if the subjects in the financial system are abstracted as network nodes, and the interactions between the subjects are abstracted as connecting lines or edges between nodes, then the entire system can be abstracted as a complex network with multiple node associations. Since network analysis describes the structure of relationships among a set of nodes and various network measures capture different aspects in a network, such as the mutual dependency among different financial subjects and then classify them, thus using the complex networks indicators, which reflect the topology and evolution of financial market networks, to study the financial contagion might provide a new way to solve this problem.

And in the context of global economic integration, people have realized that all the markets of countries, regions and industries across the world are closely linked network given the fact of the rapid contagion of financial crisis[2]. And the importance of this connectivity has become more prominent since the 2008 financial crisis. Therefore, only by combining the complex networks methods and study on the spread of financial crisis from a global perspective, can we analyze the process and path of contagion of financial crisis more deeply[3,4].

Currently how to measure the adjacent relationship among financial markets is the key factor to construct complex networks. Previous studies have showed the financial network based on the correlation is the most popular one and the correlation is mainly divided into three categories. The first method adopts the Pearson correlation coefficients to measure the network. As in Mantegna (1999)[5], Vizgunov et al. (2014)[6], Wang et al. (2015)[7], Birch et al. (2016)[8], Liu et al. (2018)[9]. The second method adopts the partial correlation coefficients to measure the network. See for example, Kenett et al. (2010; 2012a; 2012b; 2015)[10–13], Ji et al. (2018)[14] and Wang et al. (2018)[15]. Other method adopts other correlation to measure the network, such as mutual information-based network[1,16,17], connectedness-based network[18,19], cointegration-based network[20–22], and entropy-based network[23–25].

From these previous studies it can be seen that complex network has been widely used in the field of financial and economic markets and various methods have been proposed to construct networks. And generally the first two methods based on correlation coefficients which describes a kind of degree of the symmetric association between two variables are always used to construct undirected and weighted networks. However, undirected network means the interdependence between two financial markets or sectors are equal which significantly does not match the practical characteristics of economic activities[26]. Therefore, the relationship in the financial and economic framework is likely to be directed, i.e., asymmetric. Various directed and weighted networks have been used in the financial markets[20,21,24,25]. Moreover, what both Pearson correlation coefficients and partial correlation coefficients describe the linear correlation, the financial and economic market is a complex and non-linear system, however. So the coefficient correlation-based measure may not be an effective method in the field of finance[27]. Hence we need other method to measure the correlation to construct networks. As transfer entropy allows to measure the directed information flow of non-linear systems from the perspective of information flow, this may make it outperform connectedness-based and cointegration-based networks both of which describe the linear correlation, although they are directed network. So we try to combine the information theory and the complex network to study the contagion of financial crisis on real economy. And we adopt the symbolic transfer entropy based on the dynamic adaptive segmentation method proposed by Wu et al. (2013)[28], which addresses the high demand for parameters compatibility in it.

At present, most of the scholars use the original data of financial markets to construct econometric models to research the contagion of financial crisis on real economy, which may necessarily be characterized by redundant and ineffective information caused by data noise in financial markets. Especially in the current era, with the rise of the internet financial and big data, financial data rapidly begin to emerge with the blowout trend, which includes not only structured data in digital form in traditional sense but also unstructured data such as texts, images and videos. This furtherly makes the financial markets generate more and more redundant and ineffective data, leading to deviations on model estimation results. Aiming to overcome this problem, we newly propose a method to construct an econometric model with financial network indicators called higher-order information in this study instead of original data, since it can be seen that from previous studies the network indictors can capture the effective information reflecting the internal structured characteristics of financial markets, which is the key factor to eliminate the redundant and ineffective information from original data. Although there have been many academics to research the importance of networks analysis[29], however, there have been no attempts to utilize them to construct models in the global financial market outlook. Recently, there have been only a few studies that use financial indictors to construct investment strategies[30–32].

On the other hand, with the increasingly economic globalization and integration, there also have been increasingly strong spatial correlation among regions, countries, markets and industries across the world[33,34]. However, in the assumptions of the traditional econometric model, the variables are independent of each other, without spatial effects of interaction. This is seriously inconsistent with the actual characteristics of economic activity[35]. Therefore, we combine complex network and spatial econometric theory, i.e., we use the network indictor as the explanatory variable to construct the specific spatial econometric models to research the contagion of financial crisis on real economy and spatial spillover and industry aggregation effects, which not only plays the merits of network indictor, also takes the spatial effects into consideration.

Accordingly, taking the European debt crisis as the research background, we expand the model that studies the contagion of financial crisis on real economy proposed by Baur (2012)[36] to a higher-order information spatial econometric model newly proposed using network indictors as explanatory variables extracted from the directed and weighted network constructed using transfer entropy based on the dynamic adaptive segmentation method. And aiming to study from a global perspective, we choose the stock indices of financial sector and nine industry sectors of real economy (including energy, raw material, industry, consumption service, consumer goods, health and medical service, information and technology, telecommunication and public services) from US, Europe and China, respectively. In addition, we also study the financial contagion using the newly proposed spatial econometric model between global financial sector represented by Down Jones financial sector and those of the three economies during the European debt crisis period. And to compare the empirical results with the undirected network, we also construct the undirected and weighted networked based on Pearson correlation coefficients most commonly used to extract network indictors to construct the higher-order information spatial econometric model. Finally we summarized the results of the three types of contagion: the global financial sector contagion on the financial sectors of the three economies, the global financial sector contagion on the nine industry sectors of them, and the domestic financial sector contagion on the nine industry sectors of them, respectively.

Our contribution in this study is mainly two-fold: first, we adopt the symbolic transfer entropy based on the dynamic adaptive segmentation method to construct the directed and weighted complex network. And second we use the indictors extracted from the newly constructed network as the explanatory variables to construct the higher-order information spatial econometric model, which provides a new perspective for the application of the complex network methodology in the financial field.

The paper is organized as follows. Section 2 presents methodologies applied to construct the directed and weighted network and calculate whose various indictors, and the construction of the proposed spatial econometric models based on the higher-order information. Section 3 reports our empirical results. Finally, concluding remarks are stated in Section 4.

## 2. Methodology and modeling

Various methods have been proposed in the literature to study the contagion effect of financial crisis on real economy. These include GARCH model[36–38], Copula model[39], event study methodology[40], and error correction model[41]. In this paper, we firstly propose the higher-order information spatial econometric model based on the symbolic transfer entropy. This model mainly has three advantages over other estimation methods. First, the model accounts for the spatial effects presented by spatial weight matrix which have been proved to exist commonly in real world[42], financial markets are no exception[43–45], and thus it can make the estimation results more accurate. Second, the transfer entropy method fits well with the complexity and nonlinear characteristics of the financial economic system, as well as the new features of trading pattern, such as electronization and informatization. Therefore, it may probably be more appropriate and effective to measure the relationship between nodes than other correlation coefficients. Third, the model accounts for the great amount, redundancy and complexity by using the indictors extracted from the constructed network instead of original data in modeling, which may can more effectively capture the inner information of financial data and thus better reflect the structure feature of financial markets.

### 2.1 The symbolic transfer entropy based on the dynamic adaptive segmentation method

In this work, we use the symbolic transfer entropy calculated from stock indices, it is a directed measurement on information delivery among data as the edges to construct complex network. This method improves the defect on directionality of information transfer; besides, it can be utilized in nonlinear systems. This makes it accord with the practical activity characteristics and nonlinear feature of financial systems[1]. And compared with the linear correlation coefficient, Pearson correlation coefficient, Kendall correlation coefficient and mutual information, transfer entropy eliminates the interference between common historical information such as common external factors. Therefore, what is derived from transfer entropy is the statistical correlation of the source self-sequences. This property makes the method a more practical and adaptable analysis tool when studying the interrelationships between complex systems.

Transfer entropy is a method that obtains the causalities of time series based on the probability distribution, Shannon entropy and statistical method. It was first proposed by German academic Schreiber (2000)[46] based on the works of Shannon and Weaver (1949)[47] and Kolmogorov (1993)[48]. Academically speaking, it is the additional information needed to predict the system status in the situation of wrongly assuming that the transfer probability is $p(i_{t+1}|i_{t}^{\left(k\right)})$ and not $p(i_{t+1}|i_{t}^{\left(k\right)},j_{t}^{\left(h\right)})$. It has been successfully applied to biological systems which can been seen in Vicente et al. (2011)[49] and Faes et al. (2013)[50], financial markets system which can been seen in Baek et al. (2005)[51], Shi et al. (2013)[52], Li et al. (2013) [53] and Liang et al. (2014) [54] and other fields such as Lizier et al.[55] (2013), Prokopenko et al. (2013)[56] and Liu et al. (2014)[57].

In the assumption of two discrete time sequences I and J, the transfer entropy that measures the directionality information and dynamic information of systems is defined as

$$T_{J\to I}=\Sigma p(i_{t+1},i_{t}^{\left(k\right)},j_{t}^{\left(h\right)})\text{log}\frac{p(i_{t+1}|i_{t}^{\left(k\right)},j_{t}^{\left(h\right)})}{p(i_{t+1}|i_{t}^{\left(k\right)})}$$ (1)

where $i_{t}^{\left(k\right)}$ and $j_{t}^{\left(h\right)}$ denote the states of system I and system J at time t, respectively. Parameters k and h denote the time delay length of systems I and J, respectively, and are commonly set as k = h = 1, meaning that both I and J are first order Markov processes. The joint probability density function (hereafter, PDF) $p(i_{t+1},i_{t}^{\left(k\right)},j_{t}^{\left(h\right)})$ denotes the probability that $i_{t+1},i_{t}^{\left(k\right)}$ and $j_{t}^{\left(h\right)}$ are in particular states. The conditional PDF $p(i_{t+1}|i_{t}^{\left(k\right)},j_{t}^{\left(h\right)})$ and $p(i_{t+1}|i_{t}^{\left(k\right)})$ denote the probability that *i*_*t*+1_ is in a particular state when the states of $i_{t}^{\left(k\right)}$, $j_{t}^{\left(h\right)}$, and $i_{t}^{\left(k\right)}$ are uncertain.

From Eq (1) we know that the transfer entropy from I to J and that from J to I is asymmetric, and the transfer entropy from I (J) to J(I) measures the influence of system I (J) on system J(I). The larger the transfer entropy is, the greater the influence. Eq (1) can be rewritten as

$${\text{T}}_{\text{J}\to \text{I}}=\text{H}({\text{i}}_{\text{t}+\text{m}}|{\text{i}}_{\text{t}})-\text{H}({\text{i}}_{\text{t}+\text{m}}|{\text{i}}_{\text{t}},{\text{j}}_{\text{t}}),$$ (2)

where H(i_t+m_|i_t_)represents the conditional information entropy in which the uncertainty of i_t+m_ is under the condition that i_t_ has a particular value. Therefore, the transfer entropy can also be understood as the information of system I at time t+1 included by the system J which is known at time t, and is excluded from the information of system I at time t.

From what described above, it can be seen that transfer entropy not only provides a way to measure the directionality information and dynamic information between systems but can also address the relationships between nonlinear systems. In addition, in essence, the transfer entropy is defined based on the information entropy, but it improves the lack of information entropy that which cannot measure the directionality of the information transfer.

However, the transfer entropy has high demands for parameter compatibility which greatly increases the difficulty of calculation and is also sensitive to noise. To address this problem, Staniek (2008)[58] propose symbolic transfer entropy (hereafter, STE) by statically dividing the data into symbolic values, but this inevitably leads to information loss. Therefore, in this study, we adopt the way in the literature Chen et al. (2017)[59] which proposes an improved dynamic adaptive segmentation method. This effectively improve the computational complexity.

### 2.2 Indicators of the directed and weighted network based on the STE

In our work, the top 20 countries in GDP are selected as the network nodes, and the symbolic transfer entropy of aggregate stock indexes between them is taken as the edge, to construct the time-varying directed and weighted network with the sliding window technology.

For a complex network, character path length, weighted clustering coefficient, global efficiency and local efficiency are the four common indictors. The following shows the calculation method of them, in which N is the set of all the nodes in the network, and n is the number of nodes[60].

1. Character path length:
  The minimum value of the sum of weight of connection edges in all the possible paths from node i to node j in the directed weighted network is known as the shortest weighted path $d_{ij}^{\to }$ from i to j, and the reciprocal $1/d_{ij}^{\to }$ is known as the transfer efficiency from i to j, i.e., $\xi_{ij}^{\to }$, which is utilized to measure the information transfer speed. The shortest path length from node i to node j is defined as follows:
  $$d_{ij}^{\to }=\sum_{w_{ij}\in g_{i\to j}}w_{ij}$$ (3)
  where *g*_*i*→*j*_ is the directed shortest path from i to j.
  The character path length of the directed weighted network is defined as the average value of the shortest path length among all the orderly node pairs:
  $$L^{\to }=\frac{1}{n}\sum_{i\in N}\frac{\sum_{j\in N,j\neq i}d_{ij}^{\to }}{n-1}$$ (4)
2. Weighted clustering coefficient:
  Considering of the difference on the weight of the weighted network connection edges, it is needed to take the influences of related correlation degrees into consideration when calculating the clustering degree among nodes. As for the given node i, the weighted clustering coefficient is defined as follows:
  $$C^{w}{\left(i\right)}^{\to }=\frac{1}{n}\sum_{i\in N}\frac{t_{i}^{\to }}{(k_{i}^{out}+k_{i}^{in})(k_{i}^{out}+k_{i}^{in}-1)-2\sum_{j\in N}w_{ij}w_{ji}}$$ (5)
  where $t_{i}^{\to }$ is the number of directed triangles composed by node i:
  $$t_{i}^{\to }=\frac{1}{2}\sum_{j,h\in N}\left(w_{ij}+w_{ji})(w_{ih}+w_{hi})(w_{jh}+w_{hj}\right)$$ (6)
  Similar to the definition of the network character path length, the network weighted clustering coefficient WC is the average value of the weighted clustering coefficient of various nodes:
  $$WC=\frac{1}{n}\sum_{i=1}^{n}C^{w}{\left(i\right)}^{\to }$$ (7)
3. Global efficiency:
  The global efficiency of the directed weighted network is defined as the reciprocal of the shortest path length of all the orderly node pairs, i.e., the average value of the delivery efficiency $\xi_{ij}^{\to }$ from i to j:
  $$E_{glo}^{\to }=\frac{1}{n}\sum_{i\in N}E_{glo,i}^{\to }=\frac{1}{n}\sum_{i\in N}\frac{\sum_{j\in N,j\neq i}{\left(d_{ij}^{\to }\right)}^{-1}}{n-1}$$ (8)
  where $E_{glo,i}^{\to }$ is the global efficiency of the node i.
4. Local efficiency:
  In the graph theory, the subgraph of node i refers to the graph composed by all the nodes connected to the node directly. The local efficiency of the network is the average value of the global efficiency of the subgraph composed by all the nodes:
  $$E_{loc}^{\to }=\frac{1}{2n}\sum_{i\in N}\frac{\sum_{j,h\in N,j,j\neq i}\left(w_{ij}+w_{ji})(w_{ih}+w_{hi})({\left[d_{jh}^{\to }(N_{i})\right]}^{-1}+{\left[d_{hj}^{\to }(N_{i})\right]}^{-1}\right)}{(k_{i}^{out}+k_{i}^{in})(k_{i}^{out}+k_{i}^{in}-1)-2\sum_{j\in N}w_{ij}w_{ji}}$$ (9)
  where $d_{jh}^{\to }(N_{i})$ and ($d_{hj}^{\to }(N_{i})$) are the shortest path length from node j to h and from node h to j in the subgraph constituted by node i.

In modeling, before choosing the specific indictor as the explanatory variable, it is first needed to calculate the correlation coefficients between the Dow Jones financial sector and each of the ten sectors including the financial sector and the 9 real industries sectors, as well as between the four indicators and each sector. Thus, for each country/region, there are totally five kinds of average correlation coefficients, then choose the one corresponding to the biggest average as the explanatory variable. If one of the indictors is chosen, the higher-order information spatial econometric model will be constructed. Otherwise, a common spatial econometric model will be constructed.

### 2.3 Model construction and hypotheses

#### 2.3.1 Model construction

According to the GARCH model proposed by Baur (2012)[36], contagion from financial sector to real industry sector is estimated as follows:

$$R_{S,i,t}=\alpha +\beta_{1}R_{FIN,t}+\beta_{2}R_{FIN,t}D_{t}+e_{S,}{}_{i,t}$$ (10a)

$$\delta_{t}^{2}=\omega +\gamma e_{{{}_{S,}}_{i,t-1}}^{2}+\eta e_{{{}_{S,}}_{i,t-1}}^{2}d_{t-1}+\lambda \delta_{t}^{2}$$ (10b)

$$e_{S,}{}_{i,t}=\delta_{t}z_{{{}_{S,}}_{i,t}}$$ (10c)

$$Z_{S,i}\sim N(0,1)$$ (10d)

where *R*_*S*,*i*,*t*_ is the return of stock index of a specific sector of country i at time of t, *R*_*Fin*,*t*_ is the return of global financial sector portfolio at the time of t. *D*_*t*_ is a dummy variable, which is 1 when t is within the crisis period; or it is taken as 0. *β*_1_ is utilized to measure the co-movement of *R*_*Fin*,*t*_ and *R*_*S*,*i*,*t*_ during the benchmark period, i.e., the spillover effect of *R*_*Fin*,*t*_ to *R*_*S*,*i*,*t*_. *β*_2_ measures the changes on the co-movement of *R*_*Fin*,*t*_ and *R*_*S*,*i*,*t*_ during the crisis period, i.e., the changes of spillover effect of *R*_*Fin*,*t*_ to *R*_*S*,*i*,*t*_. The model is also used to analyze contagion across aggregate stock market indices. In this case S represents the sum of all sectors and is substituted by market.

Thus the model can be used to test four alternative channels of contagion: aggregate stock market contagion, financial sector contagion and real industry sector contagion spread through the global financial system or the domestic financial system. To differentiate between global and domestic contagion, Eq (10) is augmented as follows:

$$R_{S,i,t}=\alpha +\beta_{1}R_{FIN,W,t}+\beta_{2}R_{FIN,W,t}D_{t}++\theta_{1}R_{FIN,i,t}+\theta_{2}R_{FIN,i,t}D_{t}+e_{S,}{}_{i,t}$$ (11)

The Eq (11) can be used to estimate changes in the co-movement of a specific sector S (*R*_*S*,*i*,*t*_) with the global financial system (*R*_*FIN*,*W*,*t*_) or with the domestic/regional financial system (*R*_*FIN*,*W*,*t*_).

Based on the above two models, we combine the spatial econometrics and complex network, expand the contagion model described by Eqs (10) and (11) to Eqs (12) and (13) respectively, newly construct the higher-order information spatial econometric model shown as follows:

$$R_{S,i,t}=\alpha +\rho WR_{S,i,t}+\beta_{1}Pro_{FIN,W,t}+\beta_{2}Pro_{FIN,W,t}D_{t}+e_{S,}{}_{i,t}$$ (12)

$$R_{S,i,t}=\alpha +\rho WR_{S,i,t}+\beta_{1}Pro_{FIN,W,t}+\beta_{2}Pro_{FIN,W,t}D_{t}++\theta_{1}R_{FIN,i,t}+\theta_{2}R_{FIN,i,t}D_{t}+e_{S,}{}_{i,t}$$ (13)

where W is the spatial weight matrix, ρ is the spatial correlation coefficient, Pro_FIN,W,t_ is a specific network indictor. And larger absolute value of ρ indicates stronger positive/negative spatial correlation. The representation of the rest parameters are the same as those of Eqs (10) and (11). And correspondingly Eq (12) is utilized to test the contagion effects of the global financial sectors on a specific sector (financial sector or non-financial sector) of country/region i, Eq (13) is utilized to differentiate between global and domestic contagion.

To compare with the common spatial econometric model based on the original data, we also construct the following models, and the difference of them with the models proposed by Baur (2012)[36] is the addition of spatial effects.

$$R_{S,i,t}=\alpha +\rho WR_{S,i,t}+\beta_{1}R_{FIN,W,t}+\beta_{2}R_{FIN,W,t}D_{t}+e_{S,}{}_{i,t}$$ (14)

$$R_{S,i,t}=\alpha +\rho WR_{S,i,t}+\beta_{1}R_{FIN,W,t}+\beta_{2}R_{FIN,W,t}D_{t}++\theta_{1}R_{FIN,i,t}+\theta_{2}R_{FIN,i,t}D_{t}+e_{S,}{}_{i,t}$$ (15)

#### 2.3.2 Model hypotheses

Following the testing framework of Baur (2012)[36], the tests and hypotheses are given below.

Test 1: (global financial contagion of financial sector)
  Compared with tranquil period, the co-movement between the financial sector of country/region i and the global financial sector increases during the crisis period. It is assumed that the European debt crisis is triggered by the crisis of the global financial sector.
Test 2: (global financial contagion of real economy)
  Compared with tranquil period, the co-movement between the real economy sector of country/region i and the global financial sector increases during the crisis period. It is assumed that the European debt crisis is triggered by the crisis of the global financial sector.
Test 3: (domestic financial contagion of real economy)
  Compared with tranquil period, the co-movement between the real industry sectors of country/region i and the domestic financial sector increases during the crisis period. It is assumed that the domestic financial sector is the source of contagion.

The null hypothesis (*H*_0_) and alternative hypothesis (*H*_1_) of tests 1–2 are listed as follows:

*H*_0_: *β*_2_ ≤ 0 (No contagion)
*H*_1_: *β*_2_ ≤ 0 (Contagion)

The null hypothesis (*H*_0_) and alternative hypothesis (*H*_1_) of test 3 are listed as follows:

*H*_0_: *θ*_2_ ≤ 0 (No contagion)
*H*_1_: *θ*_2_ ≤ 0 (Contagion)

## 3. Empirical analysis

### 3.1 Data

The data comprises daily prices of stock index of the Dow Jones financial sector and stock indices of financial sectors for the top 20 countries in GDP (US, China, Japan, Germany, Britain, India, France, Italy, Brazil, Canada, South Korea, Spain, Australia, Russia, Mexico, Indonesia, Netherlands, Turkey, Switzerland and Saudi Arabia), and the ten sectors (including financial sector and 9 non-financial sectors: Financial, Energy, Materials, Industrials, Consumer Goods, Consumer Services, Healthcare, Information Technology, Telecommunications and Utilities) of US, Europe and China. All of them are denominated in local currency. The data is obtained from Wind database covers the period from 15 April 2008 to 31 December 2014, giving a total of 1634 observations.

Based on the following event nodes of European debt crisis: Lehman applied for bankrupt on September 15, 2008, which resulted in great impact on the economy of Greece and the whole Europe. On December 16, 2009, the rating of Greece was degraded from A- to BBB+ by Standard & Poor’s, with the rating prospect of concerted degradation. On March 7, 2011, the three major rating institutions in US continued to degrade the credit rating of Greece, and the financial crisis was deteriorated. On January 10, 2013, the European debt crisis slowed down and continued. The European debt crisis is divided into the following four stages in this article: (1) September 15, 2008 –December 8, 2009: The last period of the subprime crisis, i.e., the latency period of the European debt crisis. (2) December 9, 2009 –March 7, 2011: The European debt crisis bursted and extended to other economic entities, and financial markets of impacted economic entities showed deterioration. (3) March 8, 2011 –January 10, 2013: The European debt crisis upgraded, and extended to the real economy of the economic entities. (4) January 11, 2013 –December 31, 2014: The European crisis slowed down and continued. Considering that different financial risk contagion channels of various economic entities during the European debt crisis period are taken as the emphasis in this article, the extending period and the upgrading period; i.e., during December 9, 2009 –January 10, 2013 is set as the crisis period, and the rest time is set as the stability period.

The development level of all the sectors is represented by the daily prices of stock indices first-order logarithm difference:

$${\text{R}}_{\text{t}}=(\text{ln}\;{\text{P}}_{\text{t}}-\text{ln}\;{\text{P}}_{\text{t}-1})\times 100\text{\%}$$ (16)

where R_t_ is the return of the data of t; P_t_ and P_t-1_ are the prices on date of t and date t-1, respectively.

The summary statistics of the Dow Jones financial sector and the financial sectors of US, Europe and China during the crisis period and the whole sample period are listed in Table 1.

**Table 1:** The descriptive statistics of the daily financial sectors returns of each region during the crisis and sample period.

	USA		Europe		China		Dow Jones	
	crisis	sample	crisis	sample	crisis	sample	crisis	sample
Mean	-0.0006	-0.0002	-0.0017	-0.0003	-0.0021	-0.0003	-0.0007	0.0000
Std. dev.	0.0170	0.0285	0.0202	0.0233	0.0151	0.0207	0.0106	0.040
Skewness	-0.1765	-0.1655	-0.1070	0.2561	-0.0151	0.0291	-0.3081	-1.2032
Kurtosis	7.0181	12.0383	4.7129	7.7224	4.6638	5.9425	5.2299	19.4975
J-B	509.099	4543.292	509.0988	1253.211	86.6557	481.095	167.473	15438.262

Based on Table 1, the average of the daily return of the four financial sectors during both the crisis period and the sample period are close to zero, with certain differences on standard difference, deviation and kurtosis; especially, there are some differences on JB statistical magnitude.

### 3.2 Contagion channels, higher-order spatial spillover and industry aggregation effects

As described in Section 2.2, before constructing the contagion model to study the financial contagion on the real economy and the global financial contagion, we firstly need to determine to choose either the original data, i.e., the Dow Jones financial sector, or a specific network indictor, i.e., the higher-order information, as the explanatory variable in the above equations. Therefore, we firstly calculate the correlation coefficients between the Dow Jones financial sector and each of the ten sectors, as well as the four indicators and each of the sectors, the final results are shown as in in Tables 2, 3 and 4. And limited by the length of the article, we only show the results of correlation coefficients and all the contagion results (including the global financial contagion on the financial sectors and the financial contagion on the real economy of US, Europe and China) based on the directed and weighted network using the symbolic transfer entropy method, without showing the results of the undirected network Pearson correlation coefficients. Please contact us if need.

**Table 2:** The correlation coefficients between the Dow Jones financial sector and each sector, and between the four indicators and each sector of US.

	Energy	Basic Materials	Industrials	Consumer services	Consumer goods	Healthcare	Financial	Information Technology	Telecom.	Utilities	Mean
Length	0.436	0.611	0.438	0.481	0.498	0.600	0.481	0.658	0.523	0.617	0.534
Cluster	0.527	0.496	0.461	0.366	0.237	0.267	0.392	0.368	0.217	0.419	0.375
Global	0.568	0.669	0.632	0.673	0.466	0.501	0.468	0.702	0.483	0.728	0.589
Local	0.481	0.519	0.366	0.403	0.297	0.559	0.331	0.371	0.661	0.456	0.455
Dow	0.613	0.631	0.625	0.453	0.488	0.417	0.493	0.562	0.517	0.532	0.533

The correlation based on the undirected network using Pearson correlation coefficients are not reported. Length denotes the character path length, Cluster denotes the weighted clustering coefficient, Global and Local denote the global efficiency and local efficiency. And Dow denotes the return of Dow Jones stock index.

**Table 3:** The correlation coefficients between the Dow Jones financial sector and each sector, and between the four indicators and each sector of Europe.

	Energy	Basic Materials	Industrials	Consumer services	Consumer goods	Healthcare	Financial	Information Technology	Telecom.	Utilities	Mean
Length	0.516	0.487	0.664	0.490	0.617	0.268	0.188	0.401	0.203	0.219	0.405
Cluster	0.483	0.718	0.728	0.529	0.633	0.518	0.459	0.355	0.461	0.018	0.490
Global	0.412	0.715	0.598	0.632	0.533	0.398	0.367	0.459	0.361	0.244	0.472
Local	0.307	0.225	0.284	0.395	0.361	0.227	0.108	0.447	0.117	0.203	0.267
Dow	0.397	0.628	0.617	0.567	0.461	0.433	0.206	0.532	0.150	0.127	0.412

The correlation based on the undirected network using Pearson correlation coefficients are not reported.

**Table 4:** The correlation coefficients between the Dow Jones financial sector and each sector, and between the four indicators and each sector of China.

	Energy	Basic Materials	Industrials	Consumer services	Consumer goods	Healthcare	Financial	Information Technology	Telecom.	Utilities	Mean
Length	0.267	0.235	0.221	0.207	0.178	0.129	0.291	0.174	0.158	0.176	0.204
Cluster	0.117	0.119	0.113	0.234	0.126	0.133	0.208	0.044	0.163	0.025	0.128
Global	0.041	0.037	0.051	0.073	0.066	0.057	0.043	0.022	0.062	0.032	0.048
Local	0.016	0.011	0.006	0.026	0.012	0.018	0.021	0.032	0.021	0.015	0.018
Dow	0.109	0.112	0.203	0.128	0.114	0.121	0.030	0.034	0.216	0.020	0.109

The correlation based on the undirected network using Pearson correlation coefficients are not reported.

From Tables 2, 3 and 4, we can see although not all the average values of correlation coefficients between the network indictors and each sector are larger than that between the Dow Jones financial sector and each sector, there are at least two are larger than that from the original data for each country/region, preliminarily indicating that network indictors can better extract information of financial systems. In addition, it can be seen the network indicators with the largest average values of correlation coefficients in US, Europe and China are global efficiency, clustering coefficient and character path length, respectively. Therefore, the three network indicators will be adopted to replace the original data of Dow Jones financial sector in the following modeling by utilizing the improved higher-order information spatial econometric models represented by Eqs (12) and (13).

#### 3.2.1 Global financial contagion and higher-order spatial spillover effects

The following Tables 5 and 6 show the estimation results of the model testing for global financial sector contagion on the financial sectors of US, Europe and China based on the Eqs (14) and (12).

**Table 5:** The estimation results of the global financial sector contagion on the financial sectors across US, Europe and China based on the Eq (14).

Parameter	Europe	USA	China
ρ	0.465***	0.407*	0.203***
β_1_	0.176***	0.156***	0.153*
β_2_	0.603***	0.133***	0.081**
R^2^	0.48	0.53	0.55
Log Likelihood	4867.69	4321.27	2899.31
AIC	4.97	-5.67	-4.35
SC	-4.95	-5.63	-4.32
Contagion	C	C	C

Model: *R*_*S*,*i*,*t*_ = *α* + *ρWR*_*S*,*i*,*t*_ + *β*_1_*R*_*FIN*,*W*,*t*_ + *β*_2_*R*_*FIN*,*W*,*t*_*D*_*t*_ + *e*_*S*,*i*,*t*_,

*, **, *** represent the statistical significance at the 10%, 5% and 1% levels, respectively.

**Table 6:** The estimation results of the global financial sector contagion on the financial sectors across US, Europe and China based on the Eq (12).

Parameter	Europe	USA	China
ρ	0.573***	0.500*	0.286***
β_1_	0.203***	0.212***	0.064
β_2_	0.761*	0.226**	0.060***
R^2^	0.53	0.67	0.56
Log Likelihood	5035.00	4299.95	3467.93
AIC	-6.16	-6.09	-5.19
SC	-6.14	-6.07	-5.17
Contagion	C	C	C

The results based on the undirected network using Pearson correlation coefficients are not reported. Model: *R*_*S*,*i*,*t*_ = *α* + *ρWR*_*S*,*i*,*t*_ + *β*_1_*Pro*_*FIN*,*W*,*t*_ + *β*_2_*Pro*_*FIN*,*W*,*t*_*D*_*t*_ + *e*_*S*,*i*,*t*_;

*, **, *** represent the statistical significance at the 10%, 5% and 1% levels, respectively.

Tables 5 and 6 display the results associated with Hypotheses1, thus testing the existence of contagion from the world financial sector and the financial sectors in each country/region. Firstly, from the results we can see that the two models have the same coefficient of estimation results, indicating that the empirical results are robust. Secondly, all the spatial correlation coefficients o both the two models are significant, which indicates the introduction of spatial effects is necessary. However, according to the results of R^2^ and log likelihood, compared with the Eq (14), the newly proposed Eq (12) shows certain improvement. Meanwhile, both AIC and SC show certain reduction, illustrating the higher-order information spatial econometric model is more effective.

Moreover, we can also see that (1) Though both the ρ values of the two models are significantly larger than zero, China stands out as an example of a country whose spatial correlation is the smallest (around 0.2), the reason for this may lie in the limited degree of financial market openness, leading to relatively small spatial spillover effects. (2) As described in section 2.3, when β_2_ is statistically and significantly larger than zero, there is contagion. Therefore, the estimated β_2_ of both the two models indicate all the US, Europe and China exhibit an increased co-movement, indicating that all the financial sectors are infected by the global financial sector (i.e., the original hypothesis 1 is rejected). This is consistent with the Baur (2012)[36] and Kenourgios et al. (2014)[37]. Moreover, the Europe shows the highest linked in the crisis period (0.964), which is obtained by adding up the estimated coefficients β_1_ and β_2_. This may be because the Europe is the source area of the European sovereign debt crisis.

#### 3.2.2 The domestic financial contagion, higher-order spatial spillover effects and industry aggregation effects

Tables 7–12 display the results associated with the hypothesis 3 testing for the existence of contagion from the domestic financial sector and the real economy sectors in each country/region. The test assumes that the local financial sector is infected by the global financial system firstly, and then spreads it to the domestic real economy sectors. And Tables 7, 9 and 11 represent the estimated results of the common spatial econometric models (Eq 15), whereas Tables 8, 10 and 12 represent the estimated results of the newly proposed higher-order information spatial econometric models (Eq 13), corresponding to US, Europe and China, respectively. And limited by the length of the article, we don’t report the estimation results of the same model, i.e., the Eqs (15) and (13) testing for the global financial sector contagion on the real industry sectors of US, Europe and China, in which we assume that the global financial system has a direct impact on real economy of US and Europe. This is because the real economy firms are directly affected by the GFC since lend and borrow globally. Here is the brief description of the estimated results: Among the 9 real economy sectors, there are totally 8, expect the Utilities sector of US, 6 real economy sectors expect the sectors of Telecom, Technology and Healthcare of Europe are infected by global financial system. Whereas, for China, there is no real economy sector is infected by global financial system. This is almost consistent with the findings of Baur (2012)[36] and Kenourgios et al. (2014)[37]. And for all the equations corresponding to a specific country/region, the accuracies of Eq (12) shows significant improvement compared to those of Eq (14). Anyone who need the results, please contact us.

**Table 7:** The estimation results of the Eq (15) for testing for real economy contagion (contagion from global or domestic financial sector) of Europe.

	ρ	β_1_	β_2_	θ_1_	θ_2_	R^2^	Log Likelihood	AIC	SC	Contagion
Basic Materials	0.173***	-0.931***	0.627*	0.531**	-0.081	0.48	998.364	-1.66	-1.63	
Telecom.	0.133***	-0.229***	0.013***	0.594**	0.544	0.48	2667.1543	-1.01	-0.97	
Industrials	0.301***	0.238***	0.166*	0.411**	-0.104***	0.59	4075.71	-6.72	-6.69	
Utilities	0.116***	0.107	0.201*	0.484***	0.123	0.42	4213.902	-6.32	-6.28	
Technology	0.120***	0.236***	0.401	0.592**	-0.084*	0.51	4061.16	-6.08	-6.05	
Energy	0.151***	0.401***	0.169*	0.575**	-0.041***	0.57	4261.80	-6.31	-6.28	
Consumer services	0.105***	0.128*	0.203***	0.411***	-0.104**	0.51	4275.71	-6.51	-6.48	
Consumer goods	0.149***	-2.617*	-1.391***	0.271***	-0.035***	0.33	4543.12	-6.90	-6.87	
Healthcare	0.211***	-1.338	-2.627**	0.204*	-0.059	0.54	3863.53	-6.47	-6.44	

The results of the global financial contagion on the real economy of US, Europe and China are not reported.

Model: *R*_*S*,*i*,*t*_ = *α* + *ρWR*_*S*,*i*,*t*_ + *β*_1_*R*_*FIN*,*W*,*t*_ + *β*_2_*R*_*FIN*,*W*,*t*_*D*_*t*_ + *e*_*S*,*i*,*t*_,

*, **, *** represent the statistical significance at the 10%, 5% and 1% levels, respectively.

**Table 8:** The estimation results of the Eq (13) for testing for real economy contagion (contagion from global or domestic financial sector) of Europe.

	ρ	β_1_	β_2_	θ_1_	θ_2_	R^2^	Log Likelihood	AIC	SC	Contagion
Basic Materials	0.218***	-1.255***	0.904**	0.832**	-0.704	0.56	1112.2.3	-6.47	-6.45	
Telecom.	0.186***	-0.092***	0.048*	0.463***	0.022	0.59	4576.50	-6.86	-6.83	
Industrials	0.312***	0.302***	0.217***	0.552***	-0.176***	0.77	4487.98	-6.85	-6.82	
Utilities	0.113***	0.013	0.119**	0.477***	0.058	0.58	4346.87	-6.51	-6.48	
Technology	0.127***	0.190***	0.224	0.485***	-0.204***	0.54	4091.99	-6.13	-6.10	
Energy	0.225***	-0.057**	0.453***	0.606***	-0.210***	0.58	4238.53	-6.35	-6.32	
Consumer services	0.109***	0.090***	0.125***	0.545***	-0.240***	0.61	4347.26	-6.85	-6.82	
Consumer goods	0.166***	-0.050**	-0.232***	0.301***	-0.168***	0.56	4550.53	-6.82	-6.79	
Healthcare	0.203***	-0.004	-0.182***	0.208***	-0.043	0.65	4456.742	-6.68	-6.65	

The results of the global financial contagion on the real economy of US, Europe and China are not reported. Model: *R*_*S*,*i*,*t*_ = *α* + *ρWR*_*S*,*i*,*t*_ + *β*_1_*Pro*_*FIN*,*W*,*t*_ + *β*_2_*Pro*_*FIN*,*W*,*t*_*D*_*t*_ + + *θ*_1_*R*_*FIN*,*i*,*t*_ + *θ*_2_*R*_*FIN*,*i*,*t*_*D*_*t*_ + *e*_*S*,*i*,*t*_;

*, **, *** represent the statistical significance at the 10%, 5% and 1% levels, respectively.

**Table 9:** The estimation results of the Eq (15) for testing for real economy contagion (contagion from global or domestic financial sector) of USA.

	ρ	β_1_	β_2_	θ_1_	θ_2_	R^2^	Log Likelihood	AIC	SC	Contagion
Basic Materials	0.287***	0.416***	0.163***	0.382***	0.107	0.51	3697.21	-5.56	-5.53	
Telecom.	0.213***	0.337***	0.234	0.182***	0.135	0.48	3897.21	-6.15	-6.11	
Industrials	0.188***	0.291	0.317***	0.334	0.116	0.60	4236.87	-5.87	-5.85	
Utilities	0.139***	0.401***	-1.669*	0.156***	0.203	0.36	4009.36	-4.98	-4.95	
Technology	0.112***	0.331**	-1.993*	0.213*	0.117	0.53	4229.33	-6.25	-6.23	
Energy	0.173***	0.227**	0.162***	0.305***	0.221	0.38	3369.11	-3.66	-3.63	
Consumer services	0.199***	0.221***	0.166***	0.366***	-0.176	0.56	4563.22	-5.68	-5.66	
Consumer goods	0.181***	-0.282	-0.235***	0.306***	0.153	0.49	4663.57	-6.96	-6.94	
Healthcare	0.124***	0.165	-0.231***	0.301***	-1.183*	0.57	4331.21	-6.55	-6.53	

The results of the global financial contagion on the real economy of US, Europe and China are not reported. Model: *R*_*S*,*i*,*t*_ = *α* + *ρWR*_*S*,*i*,*t*_ + *β*_1_*R*_*FIN*,*W*,*t*_ + *β*_2_*R*_*FIN*,*W*,*t*_*D*_*t*_ + *e*_*S*,*i*,*t*_,

*, **, *** represent the statistical significance at the 10%, 5% and 1% levels, respectively.

**Table 10:** The estimation results of the Eq (13) for testing for real economy contagion (contagion from global or domestic financial sector) of Europe.

	ρ	β_1_	β_2_	θ_1_	θ_2_	R^2^	Log Likelihood	AIC	SC	Contagion from
Basic Materials	0.306***	0.293***	0.071***	0.427***	0.127	0.62	4261.11	-6.38	-6.36	
Telecom.	0.227***	0.216***	0.126	0.189***	0.151	0.59	4399.55	-6.59	-6.56	
Industrials	0.201***	0.166***	0.189**	0.447***	0.052	0.74	4686.10	-7.02	-6.99	
Utilities	0.153***	0.229***	-0.086**	0.132***	0.129	0.58	4576.93	-6.86	-6.83	
Technology	0.118***	0.167***	-0.068***	0.297***	0.098	0.64	4485.87	-6.72	-6.69	
Energy	0.167***	0.135***	0.087***	0.379***	0.092	0.53	4225.76	-6.33	-6.30	
Consumer services	0.226***	0.103***	0.117***	0.489***	-0.001	0.70	4610.65	-6.91	-6.88	
Consumer goods	0.173***	-0.004	-0.161***	0.211***	0.028	0.59	4920.13	-7.38	-7.34	
Healthcare	0.139***	0.017	-0.153***	0.277***	-0.071***	0.63	4755.28	-7.12	-7.09	

The results of the global financial contagion on the real economy of US, Europe and China are not reported. Model: *R*_*S*,*i*,*t*_ = *α* + *ρWR*_*S*,*i*,*t*_ + *β*_1_*Pro*_*FIN*,*W*,*t*_ + *β*_2_*Pro*_*FIN*,*W*,*t*_*D*_*t*_ + + *θ*_1_*R*_*FIN*,*i*,*t*_ + *θ*_2_*R*_*FIN*,*i*,*t*_*D*_*t*_ + *e*_*S*,*i*,*t*_;

*, **, *** represent the statistical significance at the 10%, 5% and 1% levels, respectively.

**Table 11:** The estimation results of the Eq (15) for testing for real economy contagion (contagion from global or domestic financial sector) of China.

	ρ	β_1_	β_2_	θ_1_	θ_2_	R^2^	Log Likelihood	AIC	SC	Contagion from
Basic Materials	0.013***	-0.166	0.236	0.512***	0.200**	0.55	3769.14	-5.15	-5.13	C**
Telecom.	0.082***	-0.311	0.258	0.481***	0.227**	0.37	3227.19	-4.36	-4.34	C**
Industrials	0.117***	0.121	0.036	0.557***	0.230**	0.58	3559.17	-6.35	-6.32	C**
Utilities	0.184***	-0.317***	0.118	0.269***	-0.198***	0.50	4361.97	-6.57	-6.55	
Technology	0.267***	-0.366	-0.218	0.446***	0.173***	0.52	3211.37	-5.17	-5.14	C***
Energy	0.106***	0.253	0.231	0.539***	0.301***	0.51	4006.97	-5.81	-8.79	C***
Consumer services	0.136***	-0.342	0.227	0.446***	-0.271***	0.57	3631.21	-5.35	-5.31	
Consumer goods	0.166***	0.338	-0.157	0.601***	-0.279	0.41	3561.25	-5.48	-5.45	
Healthcare	0.129***	-2.664	0.32	0.362***	0.115	0.39	3251.61	-4.25	-4.23	

The results of the global financial contagion on the real economy of US, Europe and China are not reported. Model: *R*_*S*,*i*,*t*_ = *α* + *ρWR*_*S*,*i*,*t*_ + *β*_1_*R*_*FIN*,*W*,*t*_ + *β*_2_*R*_*FIN*,*W*,*t*_*D*_*t*_ + *e*_*S*,*i*,*t*_,

*, **, *** represent the statistical significance at the 10%, 5% and 1% levels, respectively.

**Table 12:** The estimation results of the Eq (13) for testing for real economy contagion (contagion from global or domestic financial sector) of China.

	ρ	β_1_	β_2_	θ_1_	θ_2_	R^2^	Log Likelihood	AIC	SC	Contagion
Basic Materials	0.059***	-0.020	0.064	0.729***	0.155*	0.61	3925.79	-5.88	-5.85	C*
Telecom	0.163***	-0.010	0.010	0.649**	0.046***	0.52	3686.29	-5.52	-5.49	C***
Industrials	0.128***	0.004	0.015	0.708***	0.125***	0.67	4199.29	-6.29	-6.26	C***
Utilities	0.215***	-0.035*	0.038	0.447***	-0.147***	0.51	4315.82	-6.46	-6.43	
Technology	0.314***	-0.019	-0.001	0.631***	0.116***	0.61	3654.88	-5.47	-5.44	C***
Energy	0.188***	0.041	0.017	0.748***	0.229***	0.62	3915.03	-5.86	-5.83	C***
services	0.168***	-0.002	0.002	0.696	-0.098***	0.62	4079.33	-6.11	-6.08	
Consumer goods	0.172***	0.022	-0.032	0.526***	-0.030	0.46	3825.53	-5.73	-5.70	
Healthcare	0.132***	-0.037	0.026	0.516***	0.026	0.54	3760.68	-5.63	-5.60	

The results of the global financial contagion on the real economy of US, Europe and China are not reported. Model: *R*_*S*,*i*,*t*_ = *α* + *ρWR*_*S*,*i*,*t*_ + *β*_1_*Pro*_*FIN*,*W*,*t*_ + *β*_2_*Pro*_*FIN*,*W*,*t*_*D*_*t*_ + + *θ*_1_*R*_*FIN*,*i*,*t*_ + *θ*_2_*R*_*FIN*,*i*,*t*_*D*_*t*_ + *e*_*S*,*i*,*t*_;

*, **, *** represent the statistical significance at the 10%, 5% and 1% levels, respectively.

From the statistical results, firstly it can be seen the paired (Tables 7, 8, 9, 10, 11 and 12, corresponding to US, Europe and China respectively) of estimation results including R^2^, Loglikelihood, AIC and SC of a specific country/region obtained from the Eq (13) (the higher-order information spatial econometric model) show a significant improvement than those obtained from the Eq (15) (the common spatial econometric model), supporting the finding in Tables 5 and 6 and further indicating that replacing the original data using the network indictors is more applicable and effective. Secondly, consistent with the finding in Tables 5 and 6, all the spatial correlation coefficient ρ are significantly larger than zero, again proving the introduction of the spatial effect is necessary, and also illustrating the universality of it. Therefore, the combination of the network indictor and spatial effect proposed in our work is effective and useful.

In addition, as described in section 2.3.2, in case of this type of contagion, we should focus on the coefficient θ_2_ which represents the changes of degree of co-movement of the local financial sector and the real economy sectors during the crisis period, and a positive and statistically significant coefficient estimate θ_2_ implies the existence of contagion. So the estimation results show the developed country/region exhibit no case of local financial sector contagion on the domestic real economy sectors including both US and Europe, supporting the findings of Baur (2012)[36] and Kenourgios et al. (2014)[37], indicating that the global financial system indeed has a direct impact on the real economy in developed country/region. Whereas, China, an emerging country, there are totally 5 real economy sectors including Basic Materials, Telecom, Industrials, Technology and Energy infected by domestic financial sector. i.e., for China, it’s the local financial sector that is infected by the global financial system and spreads it to other domestic real economy sectors.

Table 13 summarizes the three different types of contagion.

**Table 13:** The summarized results of the three different types of contagion.

	Global financial sector contagion	Global financial contagion on real economy	Domestic financial contagion on real economy	Sum
USA	Contagion	8	0	8
Europe	Contagion	6	0	6
China	Contagion	0	5	5
Sum	Contagion	14	5	19

On one hand, Table 13 shows the fact that compared with the real economy sectors, there is stronger evidence for contagion in the financial sector for US, Europe and China, indicating that the financial sector is the epicenter of the crisis, supporting the findings of Baur (2012)[36] and Kenourgios et al. (2014)[37]. Meanwhile a total of 19 real economy sectors are affected, with a contagion rate of up to 70.37%, and the sectors most affected are Basic Materials (3), Industrials (3) and Energy (3) and the sectors least affected are Utilities (1) and Healthcare (1). Almost the same findings are provided by Baur (2012)[36], which indicates the industry aggregation effect.

And on the other hand, Table 13 shows the sources of the financial contagion on the real economy sectors of US, Europe and China are different. All the affected real economy sectors of both US and Europe are infected by the global financial system, whereas all the affected real economy sectors China, an emerging country, is infected by domestic financial system. i.e., the increased return co-movement of the global financial system and real economy sectors often exist in the developed country/region, whereas the increased return co-movement of the domestic financial system and real economy sectors often exist in emerging country/region. The results also indicate that compared with the listed real economy companies in emerging markets, those in developed countries/regions have stronger correlation with the global financial system, i.e., the listed real economy companies in developed markets are more vulnerable to the impact of the global financial sector. It also indicates the limited openness of China and relatively low connection degree with the global financial markets. And the empirical results illustrate the finding of previous study Kumar (2012) [61] which investigated the network property of 20 global financial indices and concluded that indices corresponding to Americas and Europe are combined together to form a cluster while the Asia/Pacific indices forms another cluster during the financial crisis. The conclusion might be connected to the different financial contagion channels concluded by this work: the industrial sectors of USA and Europe are infected by global financial system, so the two regions are combined together to form a cluster while China, belongs to Asia/Pacific area, is infected by domestic financial system not global financial system, therefore forms anther cluster. The results also support the findings of other previous studies such as Yang (2013)[62], Nobi (2014)[63]and Gidea (2017)[64], all of which indicates that the topological structure of industrial sectors network changes obviously during the financial crisis, supporting the results of our work that all the three regions are infected by the financial sector, whatever from the global or domestic financial system.

## 4. Conclusions

By combing the information theory, complex network and spatial econometrics, this paper empirically investigates the contagion effects of the European debt crisis from the financial sector to real economy sectors of US, Europe and China using a newly proposed higher-order information spatial econometric model based a time-varying and directed and weighted network. In addition, the symbolic transfer entropy based on the dynamic adaptive segmentation method is used to construct the network and the newly model uses a specific network indictor instead of the original return of the financial sector index as the explanatory variable. The purpose of the study is to examine the effectiveness and usefulness of the financial network based on the return of stock indices of top 20 countries in GDP. We test for contagion across stock markets on the global level and the domestic/regional level.

The results of the study show that the spatial effects widely exist among financial sectors and real economy sectors and the hypothesis of global financial sector contagion on a specific country/region financial sector holds for US, Europe and China, indicating the financial sector is the epicenter of the crisis. While in line with Baur (2012)[36], the global financial sector contagion on real economy sectors is evident only for US and Europe, not for China, whose affected real economy sectors are all infected by domestic financial sector. The finding illustrates that the real economy sectors in developed markets are more vulnerable to global financial system while those in emerging markets are more vulnerable to domestic financial sector. In addition, the affected real economy sectors of US, Europe and China show the aggregation effect, such as the Basic Materials, Industrials and Energy sectors in US, Europe and China are all affected during the crisis period.

Moreover, the effectiveness and usefulness of the network indictors can be confirmed based on the higher accuracies of the Eqs (12) and (13) as shown in Tables 6, 8, 10 and 12 (i.e., the higher-order information spatial econometric models) compared with the accuracies of the Eqs (14) and (15) as shown in Tables 5, 7, 9 and 11 (i.e., the common spatial econometric models) testing for the three different contagion channels. This illustrate that the network indictors may be more appropriate and effective to capture information of the financial market, a non-linear and complex system.

Our work contributes to the literature by providing a new perspective for the utilization of complex network in the financial field, using the network indictors as the explanatory variables instead of the financial sector stock index data. The study use a novel higher-order spatial econometric model in combination spatial econometrics and complex network. In addition, our findings have important implications for policy makers, investors and international organizations, such as WTO, World Bank and IMF, with taking the linkages among the non-financial sectors and the markets into account during the crisis. Especially from the results the investors can learn that holding a portfolio from various sectors is less subject to the global crisis.

Based on this model and the reported empirical findings, on one hand, the future study is to be mainly focused on utilizing financial network indicators instead of industrial sectors data to construct other financial contagion and real economy models, such as generally used financial contagion models of copula, VEC and CCA, etc. By analyzing the empirical accuracies obtained from these different models, the robustness of the proposed method could be future verified. On the other hand, the main limitation of this study is that the network indictors are only used as explanatory variables in modeling, they might be used to exhibit the topological structures of financial systems in the future, which can reveal the dynamic evolution of financial networks and then future study the contagion mechanism of financial risks from the perspective of it. In addition, we have only used the symbolic transfer entropy based method to construct the complex network, but we should develop network indictors based on other non-linear measure method for capturing various market dynamic information, such as mutual information, permutation entropy and relative entropy. We hope these limitations will be addressed in future studies.

## Supporting information

S1 Dataset The main daily data of the stock index of the Dow Jones financial sector and the financial sector and 9 major real industry sectors (energy, raw material, industry, consumption service, consumer goods, health and medical service, information and technology, telecommunication and public services) of US, Europe and China from April 15, 2008 through December 31, 2014 were obtained from the Wind database. (ZIP)
